The article "Effect of Tumor Red Blood Cell Immunity and Tumor Cell Cycle in Mice Bearing Solid Liver Cancer with Intelligent Cancer Zhongning Therapeutic Apparatus" was retracted in 2023. Reason: concerns about the peer review.

# Effect of Tumor Red Blood Cell Immunity and Tumor Cell Cycle in Mice Bearing Solid Liver Cancer with Intelligent Cancer Zhongning Therapeutic Apparatus

**DOI:** 10.1155/2021/3329800

**Published:** 2021-06-04

**Authors:** Yakun Ge, Zhehan Zhang

**Affiliations:** ^1^Institute of Biomedical Engineering, Hangzhou Dianzi University, Hangzhou 310018, Zhejiang, China; ^2^College of Pharmaceutical, Zhejiang Chinese Medical University, Hangzhou 310053, Zhejiang, China

## Abstract

People's unhealthy lifestyles, especially the number of smoking and passive smoking populations, are increasing year by year and the population is aging. With the development and progress of lung cancer cell and molecular biology, the incidence rate and mortality rate of lung cancer are increasing year by year. The existing tumor biochemotherapy has rapidly developed from preliminary research and animal research to clinical research. The smart cancer Zhongning therapeutic device can induce necrosis and apoptosis of tumor cells. The effect of treating tumors is getting more and more attention. Therefore, this article focuses on the effect of the smart cancer Zhongning therapeutic device on the tumor red blood cells and tumor cell cycle of mice with solid liver cancer. The immunological effects of the drug were discussed. Forty mice were randomly divided into high-dose group, low-dose group, 5-FU group, and model group. The effects of different treatment stages on tumor red blood cell immune function and cell cycle were recorded and evaluated, and the survival rate by multiplying the positive limit method was calculated. The model group is controlled by the exact probability method, and the Pss18.0 system is used to test the hypothesis of survival rate comparison. The experimental results showed that the tumor inhibition rate in this group was 65.8%. Compared with the 5-FU group and model group, the dose group has shown an antitumor effect and had significantly improved the tumor-bearing body's antitumor red blood cell immune function and tumor cell cycle.

## 1. Introduction

There is an inseparable relationship between the immune function of the body and the occurrence and development of tumors. When the host cells are blocked or significantly lower than the normal value, the evaluation rate should be increased, while when the tumor is growing, the immune function of tumor patients will be inhibited, which is a causal relationship. The improvement of cell cycle and tumor pathogenesis research is forming a new tumor treatment strategy. Medicine has made progress in inhibiting tumor deterioration, enhancing patients' physique, and alleviating patients' condition.

In the past 20 years, the gender and urban-rural differences in the incidence of lung cancer in China have been significantly reduced, and the age of onset has tended to be aging. At present, about 70% of lung cancer is diagnosed in an advanced stage, and the average 5-year survival rate of advanced-stage lung cancer is 15%–20%, which seriously threatens human health and increases the economic burden. After years of exploration, the treatment of lung cancer has formed a comprehensive multidisciplinary treatment, including surgical treatment, radiotherapy, chemotherapy, biologically targeted therapy, and traditional Chinese medicine. Continuous research and exploration of new methods for treating lung cancer are still the direction of our efforts. As a physical factor of nonionizing radiation, Aizhongning hyperthermia instrument has a thermal effect and nonthermal effect, which can trigger the apoptosis of nuclear cells. Many clinical medicines and animal experiments have generally confirmed that the intelligent Aizhongning treatment instrument can induce a variety of tumor cells to undergo apoptosis and preliminary exploration of related mechanisms.

Although radiotherapy combined with chemotherapy (RCT) or radiotherapy combined with EGFR blockade is more effective than radiotherapy alone, it needs to be optimized. Tinhoferd thought that the blocking of immunocheckpoint may work together with radiation, so Tinhoferd looked for the evidence of immunocheckpoint inhibitor combined with radiotherapy for SCCHN in the literature. Tinhoferd analyzed the molecular mechanism of SCCHN immune evasion, described the biological effects of radiotherapy and chemotherapy on tumor cells and immune cell microenvironment in detail, and revealed the significant interference of two treatment methods against tumor immunity. Tinhoferd's research method is highly feasible but lacks stability [1]. Rotavirus vaccines do not work well in infants in low-and middle-income countries, and intestinal microbiota is believed to affect the immune response of oral vaccines. Therefore, Twitchell established an intestinal flora (GN) pig model to study the effect of human intestinal flora (HGM) on the immune response of rotavirus vaccine and the impact of rotavirus challenge on HGM by colonizing healthy HGM (hhgm) or unhealthy HGM (uhgm) to GN pigs. Twitchell vaccinated pigs, challenged a subgroup, and evaluated the immune response and intestinal microbiota. Twitchell's research method lacks certain sample reference and its reliability is low [2]. Catastrophic antiphospholipid syndrome (APS) is characterized by the formation of multiple organ thrombus in a short period of time, which is usually related to thrombotic microangiopathy (TMA), in which the increased activation of endothelial complement in APL-positive patients plays a role in hypercoagulability. Erkan activated complement in the APS mouse model. The interaction between complement (c) 5A and its receptor C5aR leads to APL-induced inflammation, placental dysfunction, and thrombosis. The clinical study of anti-C5 monoclonal antibody in APL-positive patients is limited to a few cases. Erkan treated antiphospholipid syndrome by establishing an APS mouse model. This method is very good, but there are no data to explain it [3].

In this study, 40 mice with solid liver cancer were selected to establish the model, which was divided into four groups: high-dose group, low-dose group, 5-FU group, and model group, with 10 mice in each group. In order to further analyze the mechanism of action in the treatment of liver cancer, the antitumor effect and cell cycle of the tumor-bearing mice were recorded and observed, and the antitumor effect of the tumor-bearing mice was discussed in the direction of modern tumor immunology. Before and after the operation, the condition of mice was analyzed and compared, and SPSS18.0 system was used to study the difference of effect before and after the treatment of liver cancer.

## 2. Liver Cancer and Tumor

### 2.1. Tumor

As we all know, tumor is the result of many factors, many genes, and many mutations. Most patients with clinically confirmed tumors need to be cured with traditional Chinese medicine or a combination of traditional Chinese and Western medicine, so using traditional Chinese medicine to treat tumors has become an effective way of adjuvant treatment. In this study, we developed the formula and discussed its antitumor effect and mechanism [4, 5].

Due to the development and progress of tumor cell biology and molecular biology, the current tumor biochemical therapy has developed rapidly from preliminary research and animal research to clinical research. Biotherapy and chemotherapy of tumor biochemical therapy have been a kind of upgraded comprehensive treatment method combined with biochemical therapy. The combination can play a cumulative or synergistic effect, pay attention to the pathological type, clinical stage, location, and development trend of tumor, strengthen the tolerance of host according to the occurrence status and molecular biological characteristics of patients, and reduce the occurrence of the tumor to a great extent. Chemotherapy is recognized as one of the most advanced anticancer therapies in the world. In clinical research, most patients with liver cancer have a low tolerance to systemic chemotherapy, and alternative immunotherapy has become a research hotspot. Immunotherapy is to activate and clear tumor-specific immunity by identifying tumor-specific proteins. At present, many immunotherapies have shown antitumor immune activity, some of which have shown antitumor therapeutic effects [6, 7]. Due to the spread of health knowledge and the improvement of science and technology and people's attention to the physical examination, the detection rate of liver cancer has been increasing, and the clinical treatment of liver cancer has been paid more and more attention. Although there is no internationally recognized standard for treating liver cancer, due to the continuous expansion and breakthrough of new technologies and methods, there will be more and more advanced and reasonable targeted treatment methods for liver cancer.

### 2.2. Liver Cancer

#### 2.2.1. Liver Cancer

Liver cancer is a cancer originating from liver cells. It is a common cancer of the liver, which is caused by the mutation of liver cells in DNA. Primary liver cancer is a disease that occurs when healthy cells in the liver become abnormal in appearance and behavior. After that, cancer cells will destroy adjacent normal tissues and spread to other areas of the liver and organs outside the liver [8, 9]. There are many treatment options for liver cancer. The choice of treatment depends on the extent of cancer spread, the overall health of the liver, and the health level of the patient. Generally, CT scan and liver contrast MRI are the preferred imaging methods to detect the location and degree of blood supply of cancer. If any imaging research is inconclusive, alternative imaging or follow-up imaging research should be carried out.

#### 2.2.2. Problems in the Treatment of Liver Cancer

At present, there are many problems in the treatment of liver cancer.

#### 2.2.3. Clinical System Still Cannot Deal with Cancer

The effect of general chemotherapy on many cancer patients is very poor or almost zero. Generally speaking, the current chemotherapy system is not aimed at proliferating cells but at tumor cell-specific abnormalities. Therefore, the treatment path between model cells and tumor cells is very narrow, which leads to extremely serious side-effects of chemotherapy, such as gastrointestinal toxicity, alopecia, and myelosuppression; the treatment effect of patients and the level of jiangkang are low [5, 10]. Cancer cells are generally resistant to drugs, which makes the treatment of advanced cancer almost ineffective. Because of these problems, there is an urgent need to develop more effective long-term cancer treatment drugs.

#### 2.2.4. Cell Cycle and Cancer

Omental tumor suppressor protein (PRB) is a typical example. It changes into an important regulatory point in tumor cells. PRB regulates the process from G1 to S phase by influencing the extreme point. Because of the unusual high-frequency regulation of PRB, the abnormal operation of the PRB/E2R (transcription factor) pathway has become the standard reference for tumor cells [11]. Although E2F is an obvious target for interventional therapy, multiple factors related to PRB/E2F pathway (such as upstream CDK signal and downstream chromatin regulation) are another drug target of concern. This article proposes the minimum delay fusion path method accordingly:

(1) $$\begin{array}{c} T_{n}\left(i\right)=\delta \frac{r_{i}}{w_{i}}...\left(i\in N\right). \end{array}$$

The specific algorithm is as follows:

(2) $$\begin{array}{c} f=\left[-\frac{1}{2}\sum_{c=1}^{i}\sum_{d=1}^{i}\left(a_{c}^{*}-a_{c}\right)\left(a_{c}-a_{c}^{*}\right)Q\left(x_{c},x_{d}\right)-\vartheta \sum_{c=1}^{i}\left(a_{c}^{*}+a_{c}\right)+\sum_{c=1}^{i}b_{c}\left(a_{c}^{*}+a_{d}\right)\right]. \end{array}$$

Among them,

(3) $$\begin{array}{c} \sum_{c=1}^{i}a_{c}^{*}=\sum_{c=1}^{i}\text{ac}\;a_{c}^{*},a_{c}\in \left[0,D\right]\left(c=1,2,3,...,m\right). \end{array}$$

Among them, *D* is a normal number; this is the penalty factor. If the value of *D* is large, it means that the penalty for deviation is large. At this time, the regression function can be expressed as

(4) $$\begin{array}{c} V=\sum_{c=1}^{i}\left(a_{c}^{*}-a_{c}\right)Q\left(x_{c},x\right)+s,\\ a_{c}\in \left(0,D\right),\\ s=d_{c}-\sum_{c=1}^{i}\left(a_{c}^{*}-a_{c}\right)b\left(x_{c},x\right)+\vartheta ,\\ a_{c}^{*}\in \left(0,D\right),\\ s=d_{c}-\sum_{c=1}^{i}\left(a_{c}^{*}-a_{c}\right)b\left(x_{c},x\right)-\vartheta . \end{array}$$

Since the response variable *Y* obeys the binomial distribution, then *Y* ~ *b*(1, *π*(*X*)) can be set. At this time, *E*(*Y*)=*π*(*X*), the feasibility distribution of an observation of the sample is as follows:

(5) $$\begin{array}{c} P\left(y_{i}|X_{i}\right)=\pi {\left(X_{i}\right)}^{y_{i}}{\left[1-\pi \left(X_{i}\right)\right]}^{1-y_{i}}. \end{array}$$

Here, *X*_*i*_=[*x*_*i*1_, *x*_*i*2_,…, *x*_*in*_] *i*=1,2,…, *n*, and the maximum likelihood function of *n* sample observations is as follows:

(6) $$\begin{array}{c} L\left(\beta |X,y\right)=\prod_{i=1}^{n}{\left[\pi \left(X_{i}\right)\right]}^{y_{i}}{\left[1-\pi \left(X_{i}\right)\right]}^{1-y_{i}}. \end{array}$$

The log-likelihood function is as follows:

(7) $$\begin{array}{c} l\left(\beta \right)=\sum_{i=1}^{n}\left\{y_{i}\ln\left[\pi \left(X_{i}\right)\right]+\left(1-y_{i}\right)\left[1-\pi \left(X_{i}\right)\right]\right\}. \end{array}$$

Then, the log-likelihood function can be rewritten as follows:

(8) $$\begin{array}{c} l\left(\beta \right)=\sum_{i=1}^{n}y_{i}\beta X_{i}-\sum_{i=1}^{n}\ln\left[1+\exp\left(\beta X_{i}\right)\right], \end{array}$$

where *x*_*i*0_=1; let *f*(*β*)=*l*(*β*), then

(9) $$\begin{array}{c} \nabla f\left(\beta \right)=\frac{\partial f}{\partial \beta },\;H\left(\beta \right)=\left[\begin{array}{ccc} \frac{\partial^{2}f}{\partial \beta_{0}^{2}} & \cdots & \frac{\partial^{2}f}{\partial \beta_{0}\partial \beta_{P}}\\ \vdots & \ddots & \vdots \\ \frac{\partial^{2}f}{\partial \beta_{P}\partial \beta_{0}} & \vdots & \frac{\partial^{2}f}{\partial \beta_{P}^{2}} \end{array}\right]. \end{array}$$

### 2.3. Treatment Uncertainty

More research data are needed to find out whether the therapeutic drugs based on tumor mechanism produce drug resistance, in which tumor cells can obtain drug resistance phenotype by many different mechanisms. However, it is difficult to detect the drug resistance of inhibitors, especially in vitro, which needs to be confirmed by many studies. Similarly, if the drug resistance is judged as the obstruction of clinical medication, it can be combined with other treatment methods to reduce the disease rate. Most evidence shows that both chemosensitivity and chemoprotection (CHK2/p53) pathways of drugs can produce therapeutic effects, so drugs that change CHK1 and CHK2 can expand the scope of anticancer drugs.

## 3. Tumor RBC Immunity

### 3.1. Brief Introduction of Tumor RBC Immunity

The change of RBC immune function in tumor metastasis refers to the pathological process of tumor cells spreading from the initial site to other organs, which is a complex and multistage process. This is also the result of the interaction between tumor cells and host cells: on the one hand, the characteristics of tumor cells determine their ability to achieve the whole transfer process, that is, adhesion transfer on the surface of cell membrane and some enzymes and antigenic substances released by cells [12, 13]. On the other hand, the host's internal environment is used to determine whether to accept the metastasis of tumor cells; that is, the host's immune defense mechanism determines whether to reflect the characteristics of tumor metastasis and whether the immune system can be cleaned up. The tumor red blood cell immune process is shown in Figure 1:

Up to now, the experimental study on the immune function of red blood cells has made a more in-depth development, but there are still many problems to be clarified. The reduction of CRL is one of the causes of the tumor. The origin, performance, interaction mechanism, inhibition, and activation of CRL in tumor pathogenesis and its influence on the adhesion of RBC to tumor cells need to be studied in many aspects. At the same time, whether drugs can regulate the immune function of red blood cells to cure some diseases will become the next research field in the future.

### 3.2. Immune Function of Red Blood Cells

#### 3.2.1. Promoting Phagocytosis

The phagocytosis rate of biochemical cell immunity and granulocyte was 15%. When added to red blood cells, the phagocytosis rate doubled, and the red blood cell fragment also had the same effect. The antioxidants in red blood cells can protect the phagocytosis of neutrophils and the cytotoxic effect of oxygen free radicals released on neutrophils and increase the phagocytosis at the same time [14, 15]. Human erythrocytes can effectively enhance the phagocytosis of peripheral blood polymorphonuclear leukocytes (PMN). Under the interaction with red blood cells, the phagocytosis rate of yeast increased by about 65%. The enhancement effect of phagocytosis was different from the number of complement receptors (CRL) of red blood cells.

#### 3.2.2. Preventing Cancer Cells from Spreading

Although mature erythrocytes do not have nuclei, they initially have nuclei. CRL gene exists in all somatic nuclei but is only expressed on the membrane of erythrocytes. One of the important immune functions of red blood cell CRL is to participate in the regulation of complement system activation. It can carry antigen complement complex and antigen complement complex into the reticuloendothelial system (such as liver and spleen) and be phagocytized and destroyed by macrophages. By C3b immune adherence, cancer cells can activate the complement in peripheral blood and adhere to red blood cells by CRL, which is easily absorbed and engulfed by phagocytes. Because 93% of CRL in blood circulation exists in red blood cells, and the possibility of cancer cells meeting red blood cells in peripheral blood is 1000 times that of white blood cells, it is generally believed that C3b may play a strong role in red blood cells. It has been found that the red cell immune activity (rcla) of many diseases is decreased, while the red cell immune prevents the cancer cells from spreading through the blood circulation, which plays an important role in the antitumor immune mechanism.

#### 3.2.3. Regulating the Immune System

As an important part of the immune system, red blood cells participate in the natural immune, specific immune, and immune regulation of the human body, which are closely related to the production and end of a variety of diseases, and play a high role in tumor immunity. Red blood cells are not only an important part of natural immunity but also play a key role in specific immunity, which can directly kill tumor cells. It is an indisputable fact that RBC has an immune function. A large number of studies show that RBC also has a certain immune function. Red blood cells can adhere to tumor cells, and this kind of immune adhesion activity is mainly related to the type I complement receptor (E2CR) on red blood cells. At the same time, red blood cells can produce natural killer (NK) cell enhancers (NKEF) and significantly improve the killing activity of NK cells, and immune function plays an important role in the development of tumors. Previous studies only involved the immune system of white blood cells and often ignored the utility of red blood cells. Now, the new concept of the red blood cell immune system has opened a new direction to understanding the immune system. At present, further breakthroughs have been made in the experimental study and analysis of the relationship between the expression, mechanism, regulatory mechanism, and disease of RBC immune function.

## 4. Tumor Cell Cycle

### 4.1. Cell Cycle

Cell cycle is the basic process of cell life activities, which is the process from cell division to the next cell division. DNA synthesis and cell division are two important events in cell cycle. In evolution, cells change and form a series of regulatory mechanisms to ensure the accurate and orderly exchange of the cell cycle. There are mainly three types of molecules related to cell cycle regulation: cyclin, cyclin-dependent kinase (CDK), cyclin-dependent kinase inhibitor [16–18]. Cell cycle regulation is a complex biological process, which is related to the biological efficacy of protooncogenes and tumor suppressor genes. Many protooncogenes and tumor suppressor genes directly regulate the cell cycle and may also become the leading factor of cell cycle regulation [19]. By combining carcinogenic factors, they will cause mutation, deletion, heterotopia, amplification, and other changes and lead to an abnormal cell cycle so that abnormal cells continue to proliferate, resulting in the production of tumors. Tumor is a disease that gradually destroys the mechanism of cell cycle regulation, so it is of great significance to analyze the mechanism of cell cycle regulation and explore the mechanism of cell cycle regulation for understanding the occurrence and development of tumor and for clinical diagnosis and treatment. We have given formulas for standard calculations and evaluation standards:

(10) $$\begin{array}{c} Q=\frac{1}{2a^{2}r^{-1}}{\left(\frac{2b^{2}}{a^{2}r^{-1}}t-L\right)}^{-1}\left[a^{2}r^{-1}L^{2}+2\left(1-a^{2}\right)L\right]. \end{array}$$

Bring in the parameters and the weighting matrix *Q* to obtain the following:

(11) $$\begin{array}{c} \left(\frac{2b^{2}}{a^{2}r^{-1}}I_{x}-t\right)Q=\frac{1}{2}t^{2}+\frac{1-b^{2}}{a^{2}r^{-1}}t, \end{array}$$

which is available through the following formula:

(12) $$\begin{array}{c} Q^{2}+\frac{2\left(1+b^{2}\right)}{a^{2}r^{-1}}Q+\frac{{\left(1+b^{2}\right)}^{2}}{{\left(a^{2}r^{-1}\right)}^{2}}I_{x}={\left(Q+t+\frac{1-b^{2}}{a^{2}r^{-1}}I_{x}\right)}^{2}. \end{array}$$

Combining the correlation formula, we can obtain the following:

(13) $$\begin{array}{c} K=\frac{a}{2\text{rb}}\left[Q+t+\frac{1-b^{2}}{a^{2}r^{-1}}I_{x}-Q-\frac{1-b^{2}}{a^{2}r^{-1}}I_{x}\right]=\frac{a}{2\text{br}}t. \end{array}$$

The diversity density of the point is defined as how many positive packets are close to the point and how far the point is from the negative packet examples at a certain point. That is, as many points as possible are close to different positive packets and at the same time as far away as possible from the negative packets, the probability of the diversity density is expressed as follows:

(14) $$\begin{array}{c} \text{DD}\left(x\right)=\mathrm{Pr}\left(x=t|B_{1}^{+},B_{2}^{+},\ldots ,B_{n}^{+},B_{1}^{-},B_{2}^{-},\ldots ,B_{m}^{-}\right). \end{array}$$

Among them, *x* represents an independent point in the feature space and *t* represents a factual concept. Thus, the goal of the problem is to determine *t* by maximizing the diversity density, namely,

(15) $$\begin{array}{c} \arg\underset{x}{\max}\mathrm{Pr}\left(x=t|B_{1}^{+},B_{2}^{+},\ldots ,B_{n}^{+},B_{1}^{-},B_{2}^{-},\ldots ,B_{m}^{-}\right). \end{array}$$

The problem is transformed into a general problem of maximizing the diversity density. The problem is described as follows:

(16) $$\begin{array}{c} \arg\underset{x}{\max}\prod_{i}\mathrm{Pr}\left(x=t|B_{i}^{+}\right)\prod_{i}\mathrm{Pr}\left(x=t|B_{i}^{-}\right). \end{array}$$

### 4.2. Cell Cycle Regulation

The relationship between the principle of cell cycle regulation and tumor changes is a very valuable research field. The results show that cell proliferation, differentiation, aging, and apoptosis are all related to the cell cycle and play a role in inhibiting tumor cells. The presence of cyclin and the upregulation of MS can selectively inhibit the activity of CDK in tumor tissue, block the abnormal proliferation of tumor cells, and protect model cells, which is a new way of tumor treatment [20–22]. Almost all tumors have the characteristics of abnormal cell growth, blocked differentiation, and abnormal apoptosis caused by destroying the mechanism of cell cycle regulation. Choosing a new prescription and effective treatment plan to protect the model tissue and cause tumor cell differentiation and apoptosis, regulating the tumor cells deviating from the model cell cycle has become one of the new ways of antitumor treatment in the future. According to the characteristics of the medical system, we have improved the relevant calculation functions:

(17) $$\begin{array}{c} M=\frac{x}{\left(x+i+1\right)},\\ f\left(i\right)=x_{0}+x_{1}y_{1}+x_{2}y_{2}+x_{3}y_{3}, \end{array}$$

where *x* is the cosine similarity, *y* is the adjacent degree, *i* is the page ranking value, and 0, 1, 2, and 3 are the weight parameters.

(18) $$\begin{array}{c} W=\frac{N_{1}r_{1}{}^{2}}{2}+\frac{N_{2}r_{2}^{2}}{2}+N_{2}d_{2}^{2}+\left(\frac{N_{3}r_{3}^{2}}{2}+N_{3}d_{3}^{2}\right)*0.1+\frac{2}{3}N. \end{array}$$

The common biological feature of tumors is uncontrolled proliferation, and the main molecular mechanism is excessive cell proliferation and apoptosis caused by an abnormal cell cycle [23–25]. Cell proliferation is guaranteed by two extreme points (GL, S phase; G2, M phase). When the cell is damaged, by controlling the extreme points, the GL phase and/or G phase of the cell will be delayed, respectively, and at the same time, the cell will have time to achieve repair before replication and mitosis so as to ensure cell survival with high quality. When the damage exceeds the repair function range of the cell, it will cause apoptosis. Therefore, the regulation of the cell cycle plays an important role in maintaining genome stability in cell proliferation and apoptosis.

## 5. Experimental Design and Result Analysis

### 5.1. Experimental Design

#### 5.1.1. Materials and Instruments

1. Materials animals and tumor strains: 40 transplanted hepatoma mice, half male and half female, weighing (23 ± 1) g were used.
2. Medicine: the formula of cancerous and ICZTA is 14 g for each of 8 kinds of medicine, for example, Shandougen, zedoary turmeric, seaweed, and 4G for Glycyrrhiza, which is identified as medicinal. Grind each medicine into powder, mix 1/3 of the medicine powder into suspension, add 2/3 of the water to decoct, and take the liquid; each ml contains 1.159 g of raw medicine, which is sterilized and put it in a 3°C refrigerator for standby. A 4 mg/ml experimental solution was made up of standard saline and sealed in a 4°C refrigerator. See Table 1 for details.
3. Test Instruments

#### 5.1.2. Modeling and Grouping

1. Inoculation method and grouping: Aseptic operation, take ascites of mice bearing liver cancer, dilute it to 1 × 106/ml of tumor cells with 0.86% normal saline, inoculate 0.3 ml subcutaneously in the right armpit of each mouse, and branch the mice into model group (boiled water group), control group (5-FU group), high- and low-dose group of carcinogenic, four groups in total, half male and half female, 10 mice in each group.
2. Methods: The mice were inoculated with tumor cells for 24 hours and then used the medicine. The high-dose group and low-dose group were infused with 0.18 ml and 0.5 ml of the liquid, respectively, every day. The model group was infused with 0.4 ml of cold white boiled water every day. The control group was injected with 5-FU and 0.3 ml every other day.

#### 5.1.3. Test Index

1. Site of body constitution, site of tumor quality, and tumor inhibition rate of mice were evaluated
2. The immune function of tumor red blood cells was detected by the reference method
3. The cell cycle was analyzed by flow cytometry
4. Statistical processing method was used

In this article, we use the accurate probability method to test the hypothesis of survival rate comparison. The software used in the statistical test is the SPSS 18.0 system.

### 5.2. Analysis of Experimental Results

#### 5.2.1. Changes of Immune Function of Erythrocytes after Treatment with Cancer Cell

In order to analyze the therapeutic effect of different doses of ICZTA on mice with liver cancer, the growth quantity of erythrocytes in two groups and mice with solid liver cancer in ten days was recorded. The change trend of immune function of erythrocytes in each stage of the two groups is shown in Figure 2.

It can be seen from Figure 2 that the number of erythrocytes growing in the two groups of mice with solid liver cancer is increasing; that is to say, the immune function of the two groups is increasing during the treatment period of cancer cell, and the effect of the high-dose group is slightly better than that of the low-dose group.

At present, prolonging the survival time and improving the quality of life of cancer patients have been listed as the key indicators of tumor efficacy evaluation in the world. High-dose, long-term conventional chemotherapy is not reliable for improving the cure rate, reducing the recurrence rate, and increasing the effectiveness. The research of cancer transformation formula has brought a new path for the clinical treatment of tumor. The result is shown in Figure 3.

It can be seen from Figure 3 that the drug concentration is maintained at a certain high level, there are more coagulation necrotic tumor tissues in the drug implantation area, and the inhibitory effect of the drug is significantly higher than that of the control group. The components of the drug release slowly in the tumor area and can last longer than the edge chisel, which not only increases the action time of the drug on the tumor but also plays an extremely good role in killing or inhibiting tumor cells, greatly reduces systemic toxicity and side-effects, and prolongs the survival time of animals.

#### 5.2.2. Comparison of Immune Function of Tumor Red Blood Cells in Each Group of Mice

In order to understand the details of the immune function of erythrocytes treated by different groups of hepatoma mice and further compare and analyze the curative effect, the data of various immune functions tested are shown in Figure 4.

It can be seen from Figure 4 that many indexes of red blood cell immune function of mice treated by the high- and low-dose groups of carcinogenic are obviously superior to the other two groups. The wreath rates of erythrocytes (ETER, ATER, and DTER) in the three groups were significantly higher than that in the model group and 5-FU control group (*P* < 0.001), some of which were extremely close to or even beyond the model group.

Figure 5 shows the pictures obtained by flow cytometry of the model group, 5-FU group, low-dose group, and high-dose group.

It can be seen from Figure 5 that the number of S phase tumor cells in the high- and low-dose groups was higher than that in the model group, and the number of cells in the G2 + M phase was significantly lower than that in the model group. The DTER and ETER in the low-dose group were higher than those in the model group, and the ATER in the high-dose group was still lower than that in the model group. The three in the high-dose group were much higher than those in the model group, while the three in the 5-FU group were significantly lower than those in the model group, and the ETER and ATER were significantly different from those in the model group (*P* < 0.05).

#### 5.2.3. Solid-Phase Distribution of Tumor Cell Cycle in Each Group

In order to more accurately judge the changes of liver cancer condition and facilitate the timely adjustment of the test method, the cell cycle change trend of mouse tumor in multiple periods is shown in Figure 6.

As shown in Figure 6, the cell cycle changes of mice in the high and low treatment groups were significantly higher than those in the other two groups. The results showed that if part C of complement division interacted with the receptor with immune adhesion activity on the erythrocyte membrane, the immune efficacy of erythrocytes in the tumor-bearing body was significantly reduced, which was consistent with the results of this study; that is, DTER, ETER, and ATER in model group were significantly lower than those in model group (*P* < 0.01). However, the 5-FU group was lower than the model group, which may have side-effects on the blood system. However, the high-dose and low-dose groups were significantly higher than the model group (*P* < 0.01). Some of the effects were close to or beyond the model group to a large extent, which proved that the cancer compound could enhance the activity of erythrocytes in the tumor-bearing body.

It can be seen from Figures 7 and 8 that the natural Cr release rate of red blood cells obtained in the high- and low-dose groups was significantly lower than that of the model group and the control group, and the red blood cell activity was also significantly weaker than that of the other two groups. The difference was statistically significant (*P* < 0.01). It shows that the sensitivity of tumor cells to drugs is generally different in different periods, and drugs can specifically kill tumor cells or block cell cycle changes in different periods. If we can further explore the effect of the treatment of liver cancer and red blood cell immune function and cell cycle changes and fundamentally solve the liver cancer and tumor, it will have far-reaching significance for improving the curative effect.

#### 5.2.4. Effect on the Survival Time of Mice with Solid Liver Cancer

The therapeutic effect of ICZTA on mice with liver cancer has obvious advantages. The survival time is longer than that of the 5-FU injection Fuqiang treatment group; especially, 0.18 ml of high-dose group of ICZTA can significantly prolong the survival time of mice with solid type of liver cancer. The corresponding survival time and the number of mice in each group are shown in Figure 9.

It can be seen from Figure 9 that the mice in the high-dose group have the largest number of survival and the longest survival time, while the size group has zero. Liver cancer belongs to accumulation, flatulence, jaundice, and other categories. The pathogenesis of liver cancer is mainly internal injury, emotional change and fatigue, a variety of external factors and unreasonable diet, the decline of visceral function, the disorder of qi, blood and meridians, qi stagnation and blood stasis, phlegm turbid and qi stagnation, and toxin and heat accumulation for a long time. Therefore, the main treatment principle is to promote blood circulation, remove blood stasis, and strengthen the body by clearing away heat and detoxification. The above treatment methods are integrated into the whole mechanism, and the prescription is composed of kaempferol, zedoary turmeric, seaweed, and other drugs. It has the effect of clearing away heat, detoxifying, dispersing swelling, and relieving pain. Modern pharmacology has proved that it can not only effectively resist tumor but also enhance the immunity of the tumor-bearing body. A large number of studies have proved that many zedoary turmeric extracts can promote blood circulation and remove blood stasis, benefit qi, and relieve pain, which can be used to treat qi stagnation and blood stasis and inhibit the proliferation of tumor cells. It can cut off the deterioration of tumor cells, reduce the frequency of mitosis, and induce apoptosis of cancer cells. Seaweed has the effects of eliminating phlegm and softening, firming, and dissolving knots. Good medicine can treat accumulation. Modern research has found that its extract can inhibit cancer cells of many kinds of research animals to some extent. Its anticancer effect is closely related to the immune regulation of the body. It has been confirmed by most experiments that RBC immune system is an important part of the immune system, which can play a positive role in antitumor immune response to a large extent. Red blood cells can effectively prevent the transformation of cancer by directly adhering to tumor cells. At the same time, red blood cells can stimulate the immune efficacy of T cells, produce *β* cells to produce antibodies, and enhance the expression of the IL-2 receptor.

It can be seen from Table 2 that the relative expression of soluble Fas in the high- and low-dose groups was significantly higher than that in the model group and 5-FU group, while the relative expression of soluble Fas in the 5-FU group was lower than that in the model group. Scientific significance (*P* < 0.01) and further determination of inflammation-related factors such as IL-4, IL-10, IL-12, IFN-*γ*, and TGF-*β* in the high- and low-dose groups can be found to be low in the level of proinflammatory factors. In the model group and 5-FU group, the level of anti-inflammatory factors was higher than those in the model group and 5-FU group, and the difference was statistically significant (*P* < 0.01).

#### 5.2.5. CTFM Method to Measure the Results of Cell Traction

It can be seen from the distribution of the traction force of the mouse normal liver cells and Hepal-6 cells in Figure 10 that the traction force of the normal liver cells is more evenly distributed, with more focus points and a larger area. However, the traction force of cancer cells is unevenly distributed, and the area of focus is less than that of normal liver cells.

Comparing the displacement map of normal mouse liver cells and Hepal-6 cells in Figure 11, it is found that the area of the displacement field in the liver tumor cells is significantly reduced, and the maximum displacement is also reduced from 1.8 *μ*m to 1.1 *μ*m.

#### 5.2.6. Incidence Rate of Liver Cancer in Men and Women of Different Ages

To further analyze the development of liver cancer and the corresponding medical development trend, the incidence rate of men and women of different age groups is shown in Table 3.

According to Table 3, the incidence rate of liver cancer is increasing with age, and the incidence rate of male is higher than that of female. At present, prolonging the survival time and improving the quality of life of cancer patients have been listed as the key indicators of tumor efficacy evaluation in the world. High-dose, long-term conventional chemotherapy is not reliable for improving the cure rate, reducing the recurrence rate, and increasing the effectiveness. The research of cancer transformation formula has brought a new path for the clinical treatment of tumor. The results showed that the concentration of the drug remained at a certain high level; there were more coagulative necrotic tumor tissues in the drug implantation area, and the inhibition effect of the drug was significantly higher than that of the control group. In this experiment, the side effect of ICZTA in the treatment of liver cancer is small and the survival period is long, which shows that ICZTA is better than the traditional preparation and has a very broad and long-term application prospect in the future.

#### 5.2.7. Comparison of Antitumor Effect of Each Group

In order to directly reflect the effect of four groups on tumor treatment, the inhibition rate recorded and evaluated is shown in Table 4.

It can be seen from Table 4 that the tumor growth of mice bearing solid-type liver cancer can be effectively inhibited by the compound, and the tumor inhibition rate of high-dose group is 65.8%. In the process of cell cycle change, there are a series of regulatory mechanisms in the cell, which are used to ensure the orderly operation of the cell cycle. The process of cell proliferation is reflected in the change of the cell cycle. Tumor cells in different stages will produce different sensitive drug effects, while cancer cells are more focused on killing or blocking the change process of tumor cells in different periods. On this basis, it can inhibit the proliferation of tumor cells, and the mechanism of 5-FU ICZTA remains to be further studied. Abnormal cell proliferation caused by unregulated cell cycle regulation is an important biological feature of tumor cells. It is a key research direction to enhance the immune function of red blood cells and the relationship between the principle of cell cycle regulation and tumorigenesis. When the tumor changes, almost all tumors will destroy the abnormal cell proliferation and differentiation characteristics of the cell cycle regulation mechanism. The activation of protooncogene and the inactivation of tumor suppressor gene are the important research focus of antitumor research.

## 6. Conclusion

By analyzing the development of liver cancer and the existing problems and expounding the immune function and tumor cell cycle of red blood cells, this article shows that immune function plays an important role in tumor development. Now, the new concept of the red blood cell immune system has opened a new direction of the immune system. At present, further breakthroughs have been made in the experimental study and analysis of the relationship between the expression, mechanism, regulatory mechanism, and disease of RBC immune function. This study concentrates on the relationship between red cell immunity and cell cycle regulation, other mechanisms of tumor cell abnormality, and the latest data on cell cycle and drug discovery. It can be seen that the treatment of intelligent cancer Zhongning therapeutic can provide excellent opportunities for the design of a tumor mechanism system.

With the rapid development of electronic technology, the relationship between the cancer Zhongning therapeutic instrument and humans is getting closer and closer. Based on the intelligent cancer Zhongning therapeutic instrument, the treatment of tumors has a positive effect, low toxic side-effects, and less pain. It has become a successor to surgery, chemotherapy, and radiotherapy and another tumor therapy after biological therapy. Although the research on the nonthermal effect of the smart cancer Zhongning therapeutic instrument in treating tumors is still in the exploratory stage, there are still many controversies about its nonthermal effect mechanism on the organism. However, more and more attention and attention has been paid to research on the nonthermal effect mechanism; the in-depth research will provide more theoretical and experimental basis for the smart cancer Zhongning therapeutic instrument to be more widely used in clinical practice.

Although many scholars have done a lot of research on liver cancer, tumor red blood cells, and cell cycle and made outstanding achievements, at the same time, in terms of the limitations of this study and medical treatment and the existence of mice with solid liver cancer, there are still some problems that need to be solved in-depth. The genetic classification and syndrome differentiation of liver cancer are studied; because there is no unified treatment, it is difficult to judge the actual effect of various therapies. It is suggested that the disease be further classified and attributed accurately as soon as possible, and the standard vertebra for unified evaluation of curative effect should be unified, so that domestic scholars can study and treat cervical spondylosis; from the perspective of pathogenesis, the imbalance of dynamic and static balance of cervical spine is the key to the onset of cervical spondylosis. New drugs and more effective treatment programs are tested to protect model tissues, induce tumor cell differentiation and apoptosis, reactivate cell cycle regulation mechanism and model orbit, and ensure the growth, proliferation, and differentiation of model cells, so as to improve the cell cycle of tumor cells and return, which will provide a new direction for future cancer treatment.

## Figures and Tables

**Figure 1:** Tumor red blood cell immune process.

**Figure 2:** Growth curve of erythrocytes in high- and low-dose group.

**Figure 3:** Red blood cell growth in high- and low-dose groups: (a) low-dose group; (b) high-dose group.

**Figure 4:** Comparison of immune function of tumor red blood cells in each group of mice.

**Figure 5:** Four sets of flow cytometry analysis diagrams: (a) model group; (b) 5-FU group; (c) low-dose group; (d) high-dose group.

**Figure 6:** Solid-phase distribution of tumor cell cycle in each group of mice.

**Figure 7:** The expression of tumor red blood cell function in four groups of mice.

**Figure 8:** Red blood cell activity of four groups of mice.

**Figure 9:** Survival data and statistical test of mice after operation.

**Figure 10:** Changes of cell traction before and after hepatocellular carcinoma in mice.

**Figure 11:** Changes of displacement field before and after hepatocellular carcinoma in mice. (a) Measurement results of the displacement field of mouse liver cells. (b) Calculated result of displacement field of mouse Hepal-6 cells.

**Table 1:** List of main test instruments.

Equipment name	Instrument brand	Equipment name	Instrument brand
Biological safety cabinet	Thermo company	Automatic double pure water distiller	Asia Pacific Equipment Corporation
Constant temperature CO_2_ incubator	Thermo company	Constant temperature oven	Medical device company
Benchtop centrifuge	Thermo company	Optical microscope	Olympus
Low temperature ultracentrifuge	Hettich company	Precision electronic analytical balance	Jingke balance company
Refrigerator (4°C, −20°C)	Haier refrigerator	Constant temperature water bath	East Union

**Table 2:** Effects of tumor cells in different states on the expression of soluble Fas in mice.

Test items	Normal group	5-FU group	Low-dose group	High-dose group
Fas	0.63	0.45	0.89	0.94
IL-12	1.45	2.35	1.23	1.14
IFN-*γ*	1.59	2.13	1.32	1.07
IL-4	1.35	2.28	1.04	0.96
IL-10	1.80	2.46	1.46	1.37
TGF-*β*	1.31	2.34	1.09	0.99

**Table 3:** Incidence rate of liver cancer in different age groups.

Age	Incidence rate of male (%)	Incidence rate of Female (%)
0–25	0.01	0.01
25–45	10	6
45–65	65	55
65–85	86	75

**Table 4:** Comparison of antitumor effect of each group.

Group	Effect	Tumor inhibition rate (%)
Normal group	Low	12.1
5-FU group	Low	42.3
High-dose group	High	65.8
Low-dose group	High	62.7

## Data Availability

The data that support the findings of this study are available from the corresponding author upon reasonable request.
